# Bioinformatics Study Identified EGF as a Crucial Gene in Papillary Renal Cell Cancer

**DOI:** 10.1155/2022/4761803

**Published:** 2022-05-24

**Authors:** GenYi Qu, Hao Wang, Cheng Tang, Guang Yang, Yong Xu

**Affiliations:** ^1^Department of Urology, Zhuzhou Central Hospital, Zhuzhou 412000, China; ^2^Department of Urology, The First Affiliated Hospital, Hengyang Medical School, University of South China, Hengyang 421001, China

## Abstract

**Background:**

Due to a lack of knowledge of the disease process, papillary renal cell carcinoma (PRCC) has a dismal outlook. This research was aimed at uncovering the possible biomarkers and the underlying principles in PRCC using a bioinformatics method.

**Methods:**

We searched the Gene Expression Omnibus (GEO) datasets to obtain the GSE11151 and GSE15641 gene expression profiles of PRCC. We used the R package limma to identify the differentially expressed genes (DEGs). The online tool DAVID and ClusterProfiler package in R software were used to analyze Gene Ontology and Kyoto Encyclopedia of Genes and Genomes (KEGG) pathway dominance, respectively. The STRING database was utilized to construct the PPI network of DEGs. Using the Cytoscape technology, a protein-protein interaction (PPI) network that associated with DEGs was created, and the hub genes were identified using the Cytoscape plug-in CytoHubba. The hub genes were subjected to a Kaplan-Meier analysis to identify their correlations with survival rates.

**Results:**

From the selected datasets, a total of 240 common DEGs were identified in the PRCC, including 50 upregulated genes and 190 downregulated regulated genes. Renal growth, external exosome, binding of heparin, and metabolic processes were all substantially associated with DEGs. The CytoHubba plug-in-based analysis identified the 10 hub genes (*ALB*, *KNG1*, *C3*, *CXCL12*, *EGF*, *TIMP1*, *VCAN*, *PLG*, *LAMC1*, and *CASR*) from the original PPI network. The higher expression group of *EGF* was associated with poor outcome in patients with PRCC.

**Conclusions:**

We revealed important genes and proposed biological pathways that may be implicated in the formation of PRCC. EGF might be a predictive biomarker for PRCC and therefore should be investigated as a novel treatment strategy.

## 1. Introduction

Kidney carcinoma (RCC) affects the urinary tract. In 2018, over 175,000 RCC individuals died throughout the world, while about 400,000 reported cases were diagnosed [1]. The second most prevalent subtype of kidney cancer is papillary renal cell carcinoma (PRCC), which accounts for 15%-20% of RCC [2]. The prognoses of type I (basophilic) and type II (eosinophilic) PRCC are totally different. Patients with type I have a better prognosis than type II [3]. The majority of kidney cancer charities have been concentrated on pure cell renal cell carcinoma (ccRCC). The grade of PRCC was better than ccRCC, and their 5-year overall survival rate is much greater [4]. Surgery remains the first option of treatment options due to a lack of efficient diagnostic tools in the early stages of PRCC, a lack of knowledge of the molecular mechanism of PRCC, and PRCC's low susceptibility to radiotherapy and chemotherapy. Nevertheless, certain individuals are more likely to develop metastasis and recurrence following the surgery, culminating in a very bad outlook. Biological molecular markers for PRCC are presently unavailable. To create better screening and therapeutic options, it is critical to know the specific molecular mechanisms involved in the tumorigenesis, multiplication, and recurring of PRCC. In-depth studies on the prevalence and spread of renal papillary cancer, as well as the development of useful biological molecular indicators, will assist lead advances in the diagnosis and treatment of PRCC, thanks to the current advancement of medical science.

Microarray technology is an efficient, large-scale genetic data acquisition technology that allows the simultaneous study of the relationships between many thousands of gene expression levels and diseases and can provide insights into the mechanism of tumors. Bioinformatics is a technology that combines computational analysis and molecular biology, providing a clear direction for the study of genes. Microarray technology has been widely utilized to search for genetic variations at the genetic level over the last several years, which has allowed us to uncover specific genes, including DEGs and activities associated with PRCC [5, 6] tumorigenesis and development. The two mRNA microarray datasets from the Gene Expression Omnibus (GEO) collection were used to find significant DEGs among PRCC and normal kidney tubules in this investigation. To obtain an understanding of the molecular processes of tumorigenesis and progress, we analyzed Gene Ontology (GO) and Kyoto Encyclopedia of Genes and Genomes (KEGG) pathway analysis, followed by protein-protein interaction (PPI) network creation and then logistic regression for survival analysis. Finally, we identified 240 DEGs, and 10 hub genes were discovered, indicating that the expression level of EGF might be a predictable marker for PRCC.

## 2. Methods

### 2.1. Microarray Datasets

From the Gene Expression Omnibus database (http://www.ncbi.nlm.nih.gov/geo/), two gene expression profiling datasets (GSE11151 and GSE15641) were downloaded.

The inclusion criterion is that studies reporting the predictive markers that associated with the survival of PRCC from 2010 to 2020. The exclusion criterion is that articles having no relationships with PRCC as well as patients with PRCC that have already had radiotherapy and chemotherapy.

Yusenko et al. [5] supplied GSE11151, which was built on the Affymetrix GPL570 platform ([HGU133 Plus 2] Affymetrix Human Genome U133 Plus 2.0 Array); and Jones et al. [6] contributed GSE15641, which was built on the Affymetrix GPL96 platform ([HGU133A] Affymetrix Human Genome U133A Array). We used the affy package 12 with R language (version 3.6.1, http://r-project.org/) to process the raw data, which were subjected to background correction and data normalization using the RMA algorithm. 33 PRCC samples (19 in GSE11151 and 14 in GSE15641) and 26 matched normal tissues made up the raw data (3 in GSE11151 and 23 in GSE15641). We found that between two replicates, log2 fold enrichment of IP over input reads at detected peaks showed a Pearson correlation of approximately 0.81 to 0.86. A single sample captured a median of 78% of the peaks found in seven replicates.

### 2.2. Data Preprocessing and Identification of DEGs

The Bioconductor software package (http://www.bioconductor.org/) in R software (version 3.5.1, https://www.r-project.org/) was used to obtain the raw data and accompanying probe annotation information from the CEL file and transform it into a recognizable format. For background correction and data standardization, the Affy software package (http://www.bioconductor.org/packages/release/bioc/html/affy.html) in R was used. The DEGs between PRCC and normal samples were detected using the “limma” program (http://www.bioconductor.org/packages/release/bioc/html/limma.html). DEGs were defined as genes having an adjusted *P* value <0.05 and a |log fold change (FC)| of >1.5. Using the pheatmap package [7, 8] (http://www.bioconductor.org/packages/release/bioc/html/pheatmap.html), we utilized hierarchical clustering to qualitatively examine all DEGs from the microarray data and split them into two groups.

### 2.3. GO Enrichment Analysis

DAVID (https://davidd.ncifcrf.gov; version 6.8) is an online Bioinformatics database [9] that offers researchers a complete collection of functional annotation tools to determine the biological importance of certain genes. DAVID was used to do GO analysis, which included looking at cellular components (CC), molecular functions (MF), and biological process (BP) keywords. *P* values of less than 0.05 were deemed statistically significant.

### 2.4. KEGG Pathway Analysis

For pathway enrichment analysis, the Kyoto Encyclopedia of Genes and Genomes (KEGG) [10] (http://www.genome.jp/kegg/) was utilized. The ClusterProfiler package in R software was used to discover critical methods that are extremely near to the PPI network (http://www.bioconductor.org/packages/release/bioc/html/clusterProfiler.ht ml). *P* values of 0.05 or below were deemed statistically significant.

### 2.5. Construction of a PPI Network and Hub Gene Selection

The STRING search engine (https://string-db.org/) allows the researcher to look for interacting genes and is a biologically predictive web resource with a large number of proteins and known interaction functions [11]. DEG interactions were analyzed and evaluated using correlations between these functions and expression levels. The cut-off threshold was set at a composite score of more than 0.4. Using Cytoscape software [12], a PPI network was created based on the information from STRING (version 3.7.2). The STRING-based CytoHubba plug-in (http://apps.cytoscape.org/apps/CytoHubba) was used to identify the 10 genes with the greatest interactions as hub genes.

### 2.6. Survival Analysis of Hub Genes

The TCGA cohort (http://tcga-data.nci.nih.gov) was used to obtain expression profiles and clinical data for 289 PRCC samples. For survival analysis of the chosen hub genes, the Kaplan-Meier technique was employed, and log-rank *P* values were generated, with a log-rank *P* value of 0.05 or less than 0.05 being statistically significant.

## 3. Results

### 3.1. Identification of DEGs in PRCC

33 PRCC samples and 26 matched normal tissues were used in this investigation. Following comparing multiple profiling datasets (GSE11151 and GSE15641) with the R software's “limma” package, a total of 240 DEGs (Figures 1(a) and 1(b)) were discovered. When comparing PRCC specimens to normal samples, we found 50 upregulated genes and 190 downregulated genes. Figures 1(c) and 1(d) depict the volcano plot as well as heatmaps.

### 3.2. GO Enrichment Analysis

We used the online application tool DAVID to analyze the 240 DEGs to verify their roles. The DEGs of PRCC were mostly concentrated in renal growth, outflow, and negative inflation control, according to analysis. DEGs were primarily concentrated in the external exosome, extracellular area, extracellular area, a significant part of the plasma membrane, apical plasma membrane, basolateral plasma membrane, and blood microparticle when GO CC analysis was performed. DEGs were primarily concentrated in heparin-binding and transporter activity in a GO MF analysis.  Figure 2(a) and Table 1 show the results of the GO analysis.

### 3.3. The Enrichment of the KEGG Pathway

The ClusterProfiler package of R software was used to analyze the function of the pathways. DEGs were found to be enhanced in metabolic processes, glutathione metabolism, tyrosine metabolism, glycine, serine, threonine metabolism, antibiotic biosynthesis, glycolysis/gluconeogenesis, complement and coagulation streams, collecting duct acid secretion, fructose and mannose metabolism, arachidonic acid metabolic activity, PPAR signaling pathway, and phenylalanine metabolism.  Figure 2(b) and Table 2 show that the 13 KEGG pathways were associated with significantly deregulated DEGs.

### 3.4. Construction of a PPI Network and Selection of Top Hub Genes

Using the Cytoscape program, we created a PPI network graph based on the STRING data. Human proteins that interact with DEGs are represented as nodes in the PPI network (Figure 2(c)). Albumin (ALB) (AUC > 0.99, the single standardized mean difference (SMD) = 4.46), kininogen 1 (KNG1) (AUC = 0.91, SMD = 1.333), complement C3 (C3) (AUC = 0.88, SMD = 2.76), C-X-C motif chemokine ligand 12 (CXCL12) (AUC = 0.79, SMD = 1.01), epidermal growth factor (EGF), TIMP metallopeptidase inhibitor 1 (TIMP1) (AUC = 0.78, SMD = 0.45), versican (VCAN) (AUC = 0.76, SMD = 0.93), plasminogen (PLG) (AUC = 0.75, SMD = 1.89), laminin subunit gamma 1 (LAMC1) (AUC = 0.74, SMD = 1.83), and calcium-sensing receptor (CASR) (AUC = 0.71, SMD = 1.67) were the top ten hub genes. In Figure 2(d), the ten hub genes are shown.

### 3.5. Survival Analysis of Top Hub Genes

The clinical data of 289 PRCC samples were retrieved from the TCGA database for survival analysis. The 10 hub genes were then divided into groups based on their expression profiles, and survival studies were conducted. Higher EGF expression was associated with poor survival rate in PRCC patients among the 10 genes studied (Figure 3). The expressions of EGF in pancancers are shown in Figure 4(a) (cited from the TCGA database). In most cancers, the expression of EGF was higher than normal tissues. I have the analysis of EGF with immune cell markers such as CD8 and CD11b in TCGA database, as shown in Figure 4(b)(cited from the TCGA database). The results showed that the expression of EGF had no relationship with CD8 and CD11b.

In conclusion, the results showed that EGF was highly expressed in renal cell cancer and higher expression of EGF was related with poor outcome in patients.

## 4. Discussion

The second most prevalent kind of renal cell cancer is PRCC, which was accidentally found by B-ultrasound or CT examination during physical examination. Some patients have paraneoplastic syndromes, such as increased red blood cells, fever, hypertension, anemia, and weight loss. A few patients experience typical manifestations of renal cancer (hematuria, low back pain, and abdominal mass), and most have metastasized at diagnosis. The overall prediction of PRCC is better than that of ccRCC, but studies have shown that when PRCC invades the renal vein or inferior vena cava, the prognosis is significantly worse than that of ccRCC [13]. Due to a lack of early detection, most PRCC patients lack effective treatment options, which may contribute to the poor prognosis of patients. In recent years, various genes have indeed been implicated in the formation of PRCC [14], but the molecular mechanism of PRCC remains unknown. As a result, it is crucial to identify tumor-specific biomarkers and probable molecular pathways for PRCC, which will bring light for treatment of the disease. We may investigate the genetic differences of PRCC using tissue microarray, which has been widely utilized to find possible diagnosis and therapy targets in tumor growth and has also been shown to be a valuable way for identifying novel biomarkers in other illnesses [15, 16].

Two mRNA microarray datasets were used in this work to find significant DEGs between PRCC and normal kidney tissue. Analysis of two profiling datasets revealed a total of 240 overlapped DEGs, comprising 190 downregulated genes and 50 upregulated genes. To investigate possible DEGs interactions, we used GO and KEGG pathway enrichment analyses. The 240 DEGs were usually elevated in 12 terms, kidney advancement, efflux, low growth regulatory oversight, extracellular exosome, extracellular region, extracellular space, an integral component of the plasma membrane, apical plasma membrane, basolateral plasma membrane, blood microparticle, heparin-binding, and transporter activity, according to GO analysis. Furthermore, the 240 DEGs were highly enriched in 13 pathways, including metabolic processes and antibiotic biosynthesis, according to the KEGG pathway analysis. We built the PPI network using the STRING database, and 10 hub genes with a high level of connectivity were chosen in the PPI network, including *ALB*, *KNG1*, *C3*, *CXCL12*, *EGF*, *TIMP1*, *VCAN*, *PLG*, *LAMC1*, and *CASR*.

Albumin, encoded by ALB, is the most abundant protein in human blood. Albumin not only reflects the body's nutritional level but also reflects the body's inflammatory status. Albumin levels can be indicative of renal cancer prognosis, and patients of metastatic renal cell carcinoma with low serum albumin have a shorter progression-free survival [17, 18]. Kininogen 1 (KNG1) can inhibit angiogenesis and metastasis [19]. It is downregulated in glioma cells, where it is a hub gene [20]. KNG has been proven in studies to be a blood biomarker for colorectal cancer [21]. Overexpression of KNG1 has been shown to enhance glioma cell death and G1 cell cycle arrest, as well as limit glioma cell viability and angiogenesis [20]. KNG1 expression was reduced in PRCC in this investigation, although there was no statistically significant difference in survival. As a result, more study into the link between this gene and PRCC is required. CXCL12 is an alpha chemokine that is produced by stromal cells and is involved in hematopoietic stem cell homing as well as the development of B and T lymphocytes [22]. CXCL12 promotes tumor spread by mediating malignant cells via the endothelial vessel wall and extracellular matrix [23]. CXCL12 was shown to be a downregulated gene in this study. Low expression of CXCL12 in the tumor microenvironment has been shown to increase malignant lymphocyte metastasis, according to Ping et al. [24]. TIMP1 controls the expression of cell wall type 1-Matrix Metalloproteinase (MT1-MM) in urinary cancerous cells, which degrades extracellular matrix elements and other bioactive molecules, allowing for regulatory metastasis and cell proliferation [25]. Versican (VCAN) promotes tumor growth and metastasis. For RCC [26], VCAN has therapeutic and/or biomarker characteristics. PLG mRNA expression was downregulated in ccRCC patients, according to Schrodter et al. [27]. Patients with ccRCC who had increased PLG mRNA expression have longer overall survival, according to a second study [28]. PLG has been found as a positive predictive biomarker for advanced ovarian cancer [29], and similar findings have recently been described in advanced ovarian cancer. Calcium-sensitive receptors (CASR) have a role in malignant tumor bone metastases. CASR is a key component of RCC's bone metastasis process, and targeting CASR expression may be advantageous for individuals with bone metastatic RCC [30]. The link between RCC and the other two hub genes, C3 and TIMP1, has received little attention.

Overall survival analysis using the TCGA cohort was used to further establish the link between the 10 hub genes and PRCC survival prognosis. Only enhanced epidermal growth factor (EGF) expression was associated with a worse prognosis in patients with PRCC. Importantly, EGF is a growth factor that is expressed in a substantial proform (pro-EGF) on the cell membrane of a variety of cell types and may promote cell growth, proliferation, and differentiation by binding to the EGFR [31] receptor. EGF promoted cancers' development and spread and are linked to deregulation of the ERBB system [32, 33]. Upregulated EGF expression enhances ccRCC proliferation and migration [34], according to studies, and blocking EGF receptors is an effective therapy for ccRCC [35, 36]. EGF can also increase cancer spread by inhibiting epithelial-mesenchymal transition (EMT) [37] or influencing tumor lymphangiogenesis [38]. As a result, EGF might be a novel therapeutic target for PRCC as well as a possible predictive biomarker. The novelty of this study was to identify that EFG might be a predictor for PRCC, and this provides a novel idea for the treatment of PRCC. However, there are also limits of this study. First, we just analyze the data from online and did not have experiments to verify this opinion. Second, the mechanism underlying this is not so clarified, which needs further studies in future.

## Figures and Tables

**Figure 1:** In two profiling datasets (GSE11151 and GSE15641), a total of 240 DEGs were found, comprising (a) 50 upregulated genes and (b) 190 downregulated genes. (c) Volcano plot of DEGs in GSE11151 (cut-off criteria: |logFC| is 1.5 and adjusted *P* value is less than 0.05). (d) Heatmaps of top 50 DEGs in the GSE11151. (e) Volcano plot of DEGs in GSE15641 (cut-off criteria: |logFC| is 1.5 and adjusted *P* value is less than 0.05). (f) Heatmaps of top 50 DEGs in the GSE15641.

**Figure 2:** (a) GO enrichment analysis of significant DEGs in PRCC. GO stands for Gene Ontology; CC is for the cellular component; MF stands for molecular function, and BP stands for biological mechanism. (b) The DEGs are significantly associated with the KEGG pathway in PRCC. (c) Protein-protein interaction network of significant DEGs. (d) The top 10 hub genes were selected from the original PPI network.

**Figure 3:** The 10 discovered hub genes' predictive value for overall survival in patients with PRCC. A statistically meaningful value of *P* < 0.05 was used (a) *ALB*, (b) *KNG1*, (c) *C3*, (d) *CXCL12*, (e) *EGF*, (f) *TIMP1*, (g) *VCAN*, (h) *PLG*, (i) *LAMC1*, and (j) *CASR*).

**Figure 4:** (a) The expression of EGF in pancancers. (b) The relationship between EGF and immune markers in PRCC.

**Table 1:** Gene Ontology analysis of DEGs that are significantly deregulated in PRCC.

Category	Term	Count	%	*P* value
GOTERM_BP	GO:0001822~kidney development	10	4.21	0.004504347
GOTERM_BP	GO:0007588~excretion	9	3.79	5.07E-05
GOTERM_BP	GO:0045926~negative regulation of growth	6	2.53	0.007736575
GOTERM_CC	GO:0070062~extracellular exosome	108	45.5	3.36E-25
GOTERM_CC	GO:0005576~extracellular region	49	20.6	3.76E-05
GOTERM_CC	GO:0005615~extracellular space	47	19.8	1.17E-06
GOTERM_CC	GO:0005887~integral component of plasma membrane	44	18.5	1.35E-04
GOTERM_CC	GO:0016324~apical plasma membrane	24	10.1	5.34E-09
GOTERM_CC	GO:0016323~basolateral plasma membrane	15	6.32	1.18E-04
GOTERM_CC	GO:0072562~blood microparticle	11	4.64	0.036475753
GOTERM_MF	GO:0008201~heparin binding	13	5.48	0.002514782
GOTERM_MF	GO:0005215~transporter activity	13	5.48	0.027497033

**Table 2:** The significant DEGs that are associated with KEGG pathway analysis in PRCC.

Pathway ID	Term	Count	%	*P* value	Genes
hsa01100	Metabolic pathways	41	17.29	4.23E-04	ACOX2, TYRP1, SORD, GALNT7, ASS1, ALDOB, ADH1B, DPYS, KMO, ATP6V1B1, AGMAT, PIPOX, TPK1, ARG2, IDH2, DAO, HPD, ALDH6A1, DDC, UPB1, UGCG, FBP1, PCK2, MAN1C1, PCK1, KHK, CEL, G6PC, CYP17A1, PTGDS, HMGCS2, MGAM, HAO2, BHMT, PHGDH, ABAT, PRODH2, CYP4F3, CYP4F2, ATP6V0A4, and AOC3
hsa00410	Beta-alanine metabolism	5	2.11	0.002958924	ALDH6A1, UPB1, ABAT, DPYS, and AOC3
hsa00480	Glutathione metabolism	6	2.53	0.003078013	GSTA1, GPX1, GSTA3, GSTM3, GPX3, and IDH2
hsa00350	Tyrosine metabolism	5	2.11	0.004634999	DDC, TYRP1, ADH1B, HPD, and AOC3
hsa00260	Glycine, serine, and threonine metabolism	5	2.11	0.00685488	BHMT, PHGDH, DAO, PIPOX, and AOC3
hsa01130	Biosynthesis of antibiotics	11	4.64	0.008608567	HMGCS2, ASS1, ARG2, ALDOB, HAO2, PHGDH, IDH2, FBP1, DAO, PCK2, and PCK1
hsa00010	Glycolysis/gluconeogenesis	6	2.53	0.009865879	G6PC, ALDOB, FBP1, ADH1B, PCK2, and PCK1
hsa04610	Complement and coagulation cascades	6	2.53	0.011130489	PLAT, KNG1, C7, C3, SERPINA5, and PLG
hsa04966	Collecting duct acid secretion	4	1.68	0.015325625	CLCNKB, SLC4A1, ATP6V1B1, and ATP6V0A4
hsa00051	Fructose and mannose metabolism	4	1.68	0.02421185	KHK, SORD, ALDOB, and FBP1
hsa00590	Arachidonic acid metabolism	5	2.11	0.031301531	GPX1, PTGDS, GPX3, CYP4F3, and CYP4F2
hsa03320	PPAR signaling pathway	5	2.11	0.042066	ACOX2, FABP1, PCK2, FABP5, and PCK1
hsa00360	Phenylalanine metabolism	3	1.26	0.042891644	DDC, HPD, and AOC3

## Data Availability

The two gene expression profiling datasets (GSE11151 and GSE15641) were downloaded from the Gene Expression Omnibus database (http://www.ncbi.nlm.nih.gov/geo/). GSE11151 was contributed by Yusenko et al.; and GSE15641 was contributed by Jones et al.
